The article "Aerosols Transmit Prions to Immunocompetent and Immunodeficient Mice" was retracted in 2024. Reasons: errors in the data; errors in the images; unreliable results or conclusions; concerns about the results or conclusions.

# Aerosols Transmit Prions to Immunocompetent and Immunodeficient Mice

**DOI:** 10.1371/journal.ppat.1001257

**Published:** 2011-01-13

**Authors:** Johannes Haybaeck, Mathias Heikenwalder, Britta Klevenz, Petra Schwarz, Ilan Margalith, Claire Bridel, Kirsten Mertz, Elizabeta Zirdum, Benjamin Petsch, Thomas J. Fuchs, Lothar Stitz, Adriano Aguzzi

**Affiliations:** 1 Department of Pathology, Institute of Neuropathology, University Hospital Zurich, Zurich, Switzerland; 2 Institute of Immunology, Friedrich-Loeffler-Institut, Tübingen, Germany; 3 Department of Pathology, Clinical Pathology, University Hospital Zurich, Zurich, Switzerland; 4 Department of Computer Science, Machine Learning Laboratory, ETH Zurich, Zurich, Switzerland; University of Alberta, Canada

## Abstract

Prions, the agents causing transmissible spongiform encephalopathies, colonize the brain of hosts after oral, parenteral, intralingual, or even transdermal uptake. However, prions are not generally considered to be airborne. Here we report that inbred and crossbred wild-type mice, as well as *tg*a*20* transgenic mice overexpressing PrP^C^, efficiently develop scrapie upon exposure to aerosolized prions. NSE-PrP transgenic mice, which express PrP^C^ selectively in neurons, were also susceptible to airborne prions. Aerogenic infection occurred also in mice lacking B- and T-lymphocytes, NK-cells, follicular dendritic cells or complement components. Brains of diseased mice contained PrP^Sc^ and transmitted scrapie when inoculated into further mice. We conclude that aerogenic exposure to prions is very efficacious and can lead to direct invasion of neural pathways without an obligatory replicative phase in lymphoid organs. This previously unappreciated risk for airborne prion transmission may warrant re-thinking on prion biosafety guidelines in research and diagnostic laboratories.

## Author Summary

Prions, which are the cause of fatal neurodegenerative disorders termed transmissible spongiform encephalopathies (TSEs), can be experimentally or naturally transmitted via prion-contaminated food, blood, milk, saliva, feces and urine. Here we demonstrate that prions can be transmitted through aerosols in mice. This also occurs in the absence of immune cells as demonstrated by experiments with mice lacking B-, T-, follicular dendritic cells (FDCs), lymphotoxin signaling or with complement-deficient mice. Therefore, a functionally intact immune system is not strictly needed for aerogenic prion infection. These results suggest that current biosafety guidelines applied in diagnostic and scientific laboratories ought to include prion aerosols as a potential vector for prion infection.

## Introduction

Transmissible spongiform encephalopathies (TSEs) are fatal neurodegenerative disorders that affect humans and various mammals including cattle, sheep, deer, and elk. TSEs are characterized by the conversion of the cellular prion protein (PrP^C^) into a misfolded isoform termed PrP^Sc^ [1]. PrP^Sc^ aggregation is associated with gliosis, spongiosis, and neurodegeneration [2] which invariably leads to death. Prion diseases have been long known to be transmissible [3], and prion transmission can occur after oral, corneal, intraperitoneal (i.p.), intravenous (i.v.), intranasal (i.n.), intramuscular (i.m.), intralingual, transdermal and intracerebral (i.c.) application, the most efficient being i.c. inoculation [4], [5], [6], [7], [8], [9], [10], [11], [12]. Several biological fluids and excreta (e.g. saliva, milk, urine, blood, placenta, feces) contain significant levels of prion infectivity [13], [14], [15], [16], [17], and horizontal transmission is believed to be critical for the natural spread of TSEs [18], [19], [20], [21], [22], [23]. Free-ranging animals may absorb infectious prion particles through feeding or drinking [24], [25], and tongue wounds may represent entry sites for prions [26].

PrP^Sc^ has also been found in the olfactory epithelium of sCJD patients [27], [28]. Prion colonization of the nasal epithelium occurs in various species and with various prion strains [11], [12], [29], [30], [31], [32], [33], [34], [35], [36], [37]. In the HY-TME prion model, intranasal application is 10–100 times more efficient than oral uptake [29] and, as in many other experimental paradigms [38], [39], [40], [41], [42], [43], [44], the lymphoreticular system (LRS) is the earliest site of PrP^Sc^ deposition. A publication demonstrated transmission of chronic wasting disease (CWD) in cervidized mice via aerosols and upon intranasal inoculation [45], yet two studies reported diametrically differing results on the role of the olfactory epithelium or the LRS in prion pathogenesis upon intranasal prion inoculation [11], [12], perhaps because of the different prion strains and animal models used. These controversies indicate that the mechanisms of intranasal and aerosolic prion infection are not fully understood. Furthermore, intranasal administration is physically very different from aerial prion transmission, as the airway penetration of prion-laden droplets may be radically different in these two modes of administration.

Here we tested the cellular and molecular characteristics of prion propagation after aerosol exposure and after intranasal instillation. We found both inoculation routes to be largely independent of the immune system, even though we used a strongly lymphotropic prion strain. Aerosols proved to be efficient vectors of prion transmission in mice, with transmissibility being mostly determined by the exposure period, the expression level of PrP^C^, and the prion titer.

## Results

### Prion transmission via aerosols

Prion aerosols were produced by a nebulizing device with brain homogenates at concentrations of 0.1–20% (henceforth always indicating weight/volume percentages) derived from terminally scrapie-sick or healthy mice, and immitted into an inhalation chamber. As per the manufacturer's specifications, aerosolized particles had a maximal diameter of <10 µm, and approximately 60% were <2.5 µm [46].

Groups of mice overexpressing PrP^C^ (*tg*a*20*; n = 4–7) were exposed to prion aerosols derived from infectious or healthy brain homogenates (henceforth IBH and HBH) at various concentrations (0.1, 2.5, 5, 10 and 20%) for 10 min (Fig. 1A, Table 1). All *tg*a*20* mice exposed to aerosols derived from IBH (concentration: ≥2.5%) succumbed to scrapie with an attack rate of 100%. The incubation time negatively correlated with the IBH concentration (2.5%: n = 4, 165±54 dpi; 5%: n = 4, 131±7 dpi; 10%: n = 5, 161±27 dpi; 20%: n = 6, 133±8 dpi; *p* = 0.062, standard linear regression on standard ANOVA; Fig. 1A and F, Table 1, Table S1A).

**Figure 1:** Prion transmission through aerosols. (**A**) *tg*a*20* mice were exposed to aerosols generated from 0.1%, 2.5%, 5%, 10% or 20% prion-infected mouse brain homogenates (IBH) for 10 min. (**B**) Groups of *tg*a*20* and (**C**) CD1 mice were exposed for 1, 5 or 10 min to aerosols generated from a 20% IBH. Experiments were performed twice (different colors). (**D**) C57BL/6, (**E**) 129SvxC57BL/6, and *Prnp* ^o/o^ mice were exposed for 10 min to aerosols generated from 20% IBH. Kaplan-Meier curves describe the percentage of survival after particular time points post exposure to prion aerosols (y-axis represents percentage of living mice; x-axis demonstrates survival time in days post inoculation). Different colors and symbols describe the various experimental groups. (**F**) Jittered scatter plot of survival time against concentration of prion aerosols generated out of IBH with added linear regression fit (p = 0.0622). (**G**) Jittered scatter plot of survival time against exposure time for *tg*a*20* mice with added linear regression fit. The negative correlation between survival time and exposure time is significant (p<0.001***). (**H**) Consecutive paraffin sections of the right hippocampus of *Prnp* ^o/o^, *tg*a*20*, CD1 and C57BL/6 mice stained with HE (for spongiosis, gliosis, neuronal cell loss), SAF84 (PrP^Sc^ deposits), GFAP (astrogliosis) and Iba-1 (microglia). All animals had been exposed to aerosols generated from 20% IBH for 10 min. Scale bars: 100µm.

**Table 1:** Survival times of different mouse strains exposed to prion aerosols for various periods.

Genotype	inoculum concentr.	exposure (min)	n	attack rate	Incubation time (dpi)					
*tg*a*20*	0.1%	10	4	0/4	>300	>300	>300	>300		
*tg*a*20*	2.5%	10	4	4/4	120	121	208	219		
*tg*a*20*	5%	10	4	4/4	122	129	133	138		
*tg*a*20*	10%	10	5	5/5	124	133	161	167	191	
*tg*a*20*	20%	10	6	6/6	120	120	133	133	133	140
CD1	20%	1	3	0/3	>300	>300	>300			
CD1*	20%	1	4	2/4	202	202	>300	>300		
*tg*a*20*	20%	1	3	3/3	134	174	189			
*tg*a20*	20%	1	3	3/3	203	204	205			
CD1	20%	5	4	4/4	182	202	202	209		
CD1*	20%	5	3	3/3	202	202	202			
*tg*a*20*	20%	5	4	4/4	136	170	170	174		
*tg*a20*	20%	5	4	4/4	127	134	136	136		
CD1	20%	10	4	4/4	202	202	202	202		
CD1*	20%	10	4	4/4	202	202	211	235		
*tg*a*20*	20%	10	4	4/4	134	138	142	142		
*tg*a20*	20%	10	4	4/4	132	133	134	134		
C57BL/6	20%	10	4	4/4	164	182	188	188		
129SvxC57BL/6	20%	10	5	5/5	155	180	182	184	197	
*Prnp* ^o/o^	20%	10	3	0/3	>300	>300	>300			
newborn *tg*a*20*	20%	10	3	3/3	157	189	189			
newborn CD1	20%	10	3	3/3	211	211	211			

Upper panel: survival times of *tg*a*20* mice after 10-min exposure to aerosols generated from various concentrations of IBH. Lower panel: survival times of various mouse strains after exposure for 1, 5, or 10 min to infectious aerosols. Selected inoculations were repeated sequentially (asterisks) in order to estimate the reproducibility of these results.

*tg*a*20* mice exposed to aerosolized 0.1% IBH did not develop clinical scrapie within the observational period (n = 4; experiment terminated after 300 dpi), yet displayed brain PrP^Sc^ indicative of subclinical prion infection (Fig. 1A and 2A). In contrast, control *tg*a*20* mice (n = 4) exposed to aerosolized HBH did not develop any recognizable disease even when kept for ≥300 dpi, and their brains did not exhibit any PrP^Sc^ in histoblots and Western blots (data not shown).

**Figure 2:** PrP^Sc^ deposition in brains of mice infected with prion aerosols and profiling of *NSE-PrP* mice. (**A**) Western blot analysis of brain homogenates (10%) from terminal or subclinical *tg*a*20* mice exposed to aerosols from 20% or 0.1% IBH for 10 min. PK+ or −: with or without proteinase K digest; kDa: Kilo Dalton. (**B–C**): Western blot analyses of brain homogenates from *tg*a*20* (**B**) or CD1 (**C**) mice exposed to prion aerosols from 20% IBH. (**D**) Histoblot analysis of brains from mice exposed to prion aerosols. Brains of *tg*a*20* mice challenged with aerosolized 10% (middle panel) or 20% (right panel) IBH showed deposits of PrP^Sc^ in the cortex and mesencephalon. Because the brain of a *Prnp* ^o/o^ mouse showed no signal (left panel), we deduce that the signal in the middle and right panels represents local prion replication. (**E**) Histopathological lesion severity score analysis of 5 brain regions depicted as radar plots [51] (astrogliosis, spongiform change and PrP^Sc^ deposition) derived from *tg*a*20*, CD1, C57BL/6 and 129SvxC57BL/6 mice exposed to prion aerosols. Numbers correspond to the following brain regions: (1) hippocampus, (2) cerebellum, (3) olfactory bulb, (4) frontal white matter, (5) temporal white matter. (**F**) Histopathological lesion severity score of 5 brain regions shown as radar blot (astrogliosis, spongiform change and PrP^Sc^ deposition) of i.c. prion inoculated *tg*a*20*, CD1, C57BL/6 and 129SvxC57BL/6 mice. (1) hippocampus, (2) cerebellum, (3) olfactory bulb, (4) frontal white matter, (5) temporal white matter. (**G**) Survival curve and (**H**) lesion severity scores of *NSE-PrP* mice exposed to a 20% aerosolized IBH for 10 min. (**I**) Histological and immunohistochemical characterization of scrapie-affected hippocampi of *NSE-PrP* mice after exposure to aerosolized 20% IBH. Stain legend as in Fig. 1H. Scale bar: 100µm.

In the above experiments, and in all experiments described in the remainder of this study, all PrP-expressing (*tg*a*20* and WT) mice diagnosed as terminally scrapie-sick were tested by Western blot analysis and by histology: all were invariably found to contain PrP^Sc^ in their brains (Fig. 2) and to display all typical histopathological features of scrapie including spongiosis, PrP deposition and astrogliosis (Fig. 1H).

### Correlation of exposure time to prion aerosols and incubation period

We then sought to determine the minimal exposure time that would allow prion transmission via aerosols (Fig. 1B, Table 1). *tg*a*20* mice were exposed to aerosolized IBH (20%) for various durations (1, 5 or 10 min) in two independent experiments. Surprisingly, an exposure time of only 1 min was found to be sufficient to induce a 100% scrapie attack rate. Longer exposures to prion-containing aerosols strongly correlated with shortened incubation periods (Fig. 1B and G, Table 1, Table S1A and B).

In order to test the universality of the above results, we examined whether aerosols can transmit prions to various mouse strains (CD1, C57BL/6; 129SvxC57BL/6) expressing wild-type (wt) levels of PrP^C^. CD1 mice were exposed to aerosolized 20% IBH in two independent experiments (Fig. 1C, Table 1). After 5 or 10-min exposures, all CD1 mice succumbed to scrapie whereas shorter exposure (1 min) led to attack rates of 0–50% [1 min exposure (first experiment): scrapie in 0/3 mice; 1 min exposure (second experiment): 2/4 mice died of scrapie at 202±0 dpi; 5 min (first experiment): n = 4, attack rate 100%, 202±12 dpi; 5 min (second experiment): n = 3, attack rate 100%, 202±0 dpi; 10 min (first experiment): n = 4, attack rate 100%, 202±0 dpi; 10 min (second experiment): n = 4, attack rate 100%, 206±16 dpi]. In CD1 mice exposed to prion-containing aerosols for longer intervals, we detected a trend towards shortened incubation times which did not attain statistical significance (Table S1A and S1B).

We also investigated whether C57BL/6 or 129SvxC57BL/6 mice would succumb to scrapie upon exposure to prion aerosols (Fig. 1D and E, Table 1). A 10 min exposure time with a 20% IBH led to an attack rate of 100% (C57BL/6: 10 min: n = 4; 185±11 dpi; 129SvxC57BL/6: n = 5; 10 min: 182±15 dpi). Control *Prnp* ^o/o^ mice (129SvxC57BL/6 background; n = 3) were resistant to aerosolized prions (20%, 10 min) as expected (Fig. 1E and H, Table 1).

### Incubation time and attack rate depends on PrP^C^ expression levels

When *tg*a*20* mice were challenged for 10 min, variations in the concentration of aerosolized IBH had a barely significant influence on survival times (*p* = 0.062; Fig. 1F), whereas variations in the duration of exposure of *tg*a*20* mice affected their life expectancy significantly (*p*<0.001; Fig. 1G). Furthermore *tg*a*20* mice, which express 6–9 fold more PrP^C^ in the central nervous system (CNS) than wt mice [46], [47], [48], succumbed significantly earlier to scrapie upon prion aerosol exposure for 10 min (20%) (*tg*a*20* mice: 134±4 dpi; CD1 mice: 202±12 dpi, *p*<0.0001; C57BL/6 mice: 185±11 dpi, *p* = 0.003; 129SvxC57BL/6 mice: 182±15 dpi, *p* = 0.003; Fig. 1B–E, Fig. S1, Table S1A and S1C). Incubation time was prolonged and transmission was less efficient in CD1 mice than in *tg*a*20* mice after a 1 min exposure to prion aerosols (20%). The variability of incubation times between CD1 mice was low (1^st^ vs. 2^nd^ experiment with 5-min exposure: *p* = 0.62, 1^st^ vs. 2^nd^ experiment with 10-min exposure: *p* = 0.27; Fig. 1C, Table 1). This suggests that 1 min exposure of CD1 mice to prion aerosols (20%) suffices for uptake of ≤1LD50 infectious units. This finding underscores the importance of PrP^C^ expression levels not only for the incubation time but also for susceptibility to infection and neuroinvasion upon exposure to aerosols. Histoblot analyses confirmed deposition of PrP^Sc^ in brains of *tg*a*20* mice exposed to prion aerosols derived from 10% or 20% IBH, whereas no PrP^Sc^ was found in brains of *Prnp* ^o/o^ mice exposed to prion aerosols (Fig. 2D).

We then performed a semiquantitative analysis of the histopathological lesions in the CNS. The following brain regions were evaluated according to a standardized severity score (astrogliosis, spongiform change and PrP^Sc^ deposition; [49]): hippocampus, cerebellum, olfactory bulb, frontal white matter, and temporal white matter. Scores were compared to those of mice inoculated i.c. with RML (Fig. 2E and F). Lesion profiles of terminally scrapie-sick mice (*tg*a*20*, CD1, C57BL/6 and 129SvxC57BL/6) infected i.c. or through aerosols were similar irrespectively of genetic background or PrP^C^ expression levels (Fig. 2E and F), with CD1 and 129SvxC57BL/6 hippocampi and cerebella displaying only mild histological and immunohistochemical features of scrapie regardless of the route of inoculation.

We attempted to trace PrP^Sc^ in the nasopharynx, the nasal cavity or various brain regions early after prion aerosol infection (1–6 hrs post exposure) and at various time points after intranasal inoculations (6, 12, 24, 72, 144 hrs, 140 dpi, and terminally) with various methods including Western blot, histoblot and protein misfolding analyses. However, none of these analyses detected PrP^Sc^ shortly after exposure to prion aerosols (6–72 hrs post prion aerosol exposure) whereas at 140 dpi or terminal stage PrP^Sc^ was detected by all of these methods (Fig. S2; data not shown).

### PrP^C^ expression on neurons allows prion neuroinvasion upon infection with prion aerosols

We then investigated whether PrP^C^ expression in neurons would suffice to induce scrapie after exposure to prions through aerosols. *NSE-PrP* transgenic mice selectively express PrP^C^ in neurons and if bred on a *Prnp* ^o/o^ background (*Prnp* ^o/o^/*NSE-PrP*) display CNS-restricted PrP expression levels similar to wt mice [50].

*Prnp* ^o/o^/*NSE-PrP* (henceforth referred to as *NSE-PrP*) mice were exposed to prion aerosols (20% homogenate; 10 min). All *NSE-PrP* mice succumbed to terminal scrapie (216±8 dpi; n = 4; Fig. 1E, 2G, Table 1), although incubation times were significantly longer than those of wt 129SvxC57BL/6 mice (180±15 dpi; n = 5; *p* = 0.004). Histology and immunohistochemistry confirmed scrapie in *NSE-PrP* brains (Fig. 2H and I). Histopathological lesion severity score analysis (see above) revealed a lesion profile roughly similar to that of control 129SvxC57BL/6 mice (Fig. 2E, H). More severe lesions were observed in *NSE-PrP* cerebella whereas olfactory bulbs were less affected.

Real time PCR analysis revealed 2–4 transgene copies per *Prnp* allele in *Prnp* ^o/o^ */NSE-PrP* mice.

A detailed quantitative analysis of PrP^C^ expression levels at various sites of the CNS was performed by comparing the signals obtained by blotting various amounts of protein from *NSE-PrP*, wt and *tg*a*20* tissues (Fig. S3). A value of 100 was arbitrarily assigned to expression of PrP^C^ in wt tissues; olfactory epithelia of *tg*a*20* and *NSE-PrP* mice expressed ≥350 and ∼30, respectively (Fig. S3A). In olfactory bulbs, *tg*a*20* and *NSE-PrP* mice expressed ≥150 and 30, respectively (Fig. S3B). In brain hemispheres *tg*a*20* and *NSE-PrP* mice expressed >250 and >150, respectively (Fig. S3C). Therefore, *NSE-PrP* mice expressed somewhat more PrP^C^ than wt mice in brain hemispheres, but somewhat less in olfactory bulbs and olfactory epithelia.

### Aerosolic prion infection is independent of the immune system

In many paradigms of extracerebral prion infection, efficient neuroinvasion relies on the anatomical and physiological integrity of several immune system components [40], [42], [43], [44]. To determine whether this is true for aerosolic prion challenges, we exposed immunodeficient mouse strains to prion aerosols. This series of experiments included *JH* ^−/−^ mice, which selectively lack B-cells, and *γ_C_Rag2* ^−/−^ mice which are devoid of mature B-, T- and NK-cells (Fig. 3A). Upon exposure to prion aerosoIs (20% IBH; exposure time 10 min) both *JH* ^−/−^ and *γ_C_Rag2* ^−/−^ mice succumbed to scrapie with a 100% attack rate (*JH* ^−/−^: n = 6, 181±21 dpi; *γ_C_Rag2* ^−/−^: n = 11, 185±41 dpi, *p* = 0.65). The incubation times were not significantly different to those of C57BL/6 wt mice exposed to prion aerosols (*JH* ^−/−^ mice: *p* = 0.9; *γ_C_Rag2* ^−/−^ mice: *p* = 0.7).

**Figure 3:** Prion transmission through aerosols in immunocompromised mice. Survival curves, lesion severity score analysis (radar plots), and representative histopathological micrographs of mice with genetically or pharmacologically impaired components of the immune system (*JH* ^−/−^, *γ_C_Rag2* ^−/−^ **A**),129Sv mice treated with LTβR-Ig or with muIgG (**B**), *and LT*β*R* ^−/−^, and *CD40* ^−/−^ mice (**C**). All mice were exposed for 10 min to aerosolized 20% IBH. Stain code: HE (spongiosis, gliosis, neuronal cell loss), SAF84 (PrP^Sc^ deposits), GFAP (astrogliosis) and Iba-1 (microglial activation) as in Fig. 1H. Scale bars: 100µm.

Histological and immunohistochemical analyses confirmed scrapie in all clinically diagnosed mice. Lesion severity score analyses (Fig. 3A and 3E) showed that *JH* ^−/−^ and *γ_C_Rag2* ^−/−^ mice had lower profile scores in cerebella and higher scores in hippocampi and frontal white matter than C57BL/6 mice. Slightly higher scores in temporal white mater areas and the thalamus could be detected in *JH* ^−/−^ and *γ_C_Rag2* ^/−/−^ mice, whereas *γ_C_Rag2* ^−/−^ mice showed lower scores in olfactory bulbs. Consistently with several previous reports, *γ_C_Rag2* ^−/−^ mice (n = 4) did not succumb to scrapie after i.p. prion inoculation (100µl RML6 0.1% 6 log LD50) even when exposed to a prion titer that was twice higher than that used for intranasal inoculations (data not shown).

Depending on the exposure time and the IBH concentration, *tg*a*20* mice developed splenic PrP^Sc^ deposits. In contrast, none of the scrapie-sick JH^−/−^, LTβR^−/−^ and *γ_C_Rag2* ^−/−^ mice displayed any splenic PrP^Sc^ on Western blots and/or histoblots (Fig. S4A–D) despite copious brain PrP^Sc^.

### Aerosol infection is independent of follicular dendritic cells

Follicular dendritic cells (FDCs) are essential for prion replication within secondary lymphoid organs and for neuroinvasion after i.p. or oral prion challenge [42], [44], [51]. Lymphotoxin beta receptor-Ig fusion protein (LTβR-Ig) treatment in C57BL/6 mice causes dedifferentiation of mature FDCs, resulting in reduced peripheral prion replication and neuroinvasion upon extraneural (e.g. intraperitoneal or oral) prion inoculation [52], [53]. We therefore investigated whether FDCs are required for prion replication after challenge with prion aerosols. C57BL/6 mice were treated with LTβR-Ig or nonspecific pooled murine IgG (muIgG) before and after prion challenge (−7, 0, and +7 days) (Fig. 3B). The effects of the LTβR-Ig treatment were monitored by Mfg-E8^+^/FDC-M1^+^ staining for networks of mature FDCs in lymphoid tissue. This analysis revealed a complete loss of Mfg-E8^+^/FDC-M1^+^ networks at the day of prion exposure and at 14 dpi (data not shown).

LTβR-Ig treatment and dedifferentiation of FDCs did not alter incubation times upon aerosol prion infection (LTβR-Ig: n = 3, attack rate 100%, 184±0 dpi; muIgG: n = 3, attack rate 100%, 184±0 dpi) (Fig. 3B, Table 2). The diagnosis of terminal scrapie was confirmed by histological and immunohistochemical analyses in all clinically affected mice (Fig. 3B; data not shown). Histopathological lesion severity scoring revealed that LTβR-Ig treated C57BL/6 mice displayed a higher score in all regions investigated than untreated C57BL/6 mice upon challenge with prion aerosols (20% IBH; 10 min) (Fig. 2E and 3B). We found slightly less severe scores in the olfactory bulbs of C57BL/6 mice treated with muIgG than in untreated C57BL/6 mice upon challenge with prion aerosols (Fig. 2E and 3B), and a slightly higher score in the temporal white matter (exposure to 20% aerosol for 10 min; Fig. 2E and 3B).

**Table 2:** Survival of mouse strains exposed to prion aerosols (upper panel) or intranasal administered prions (lower panel).

Genotype	n	Attack rate	Survival (dpi)										
**Aerosol (20% IBH)**													
NSE-Prp	4	4/4	211	211	213	227							
JH^−/−^	6	6/6	140	184	184	188	190	198					
γ_C_Rag2^−/−^	11	11/11	121	134	141	165	169	187	224	224	224	224	227
C57BL/6 treated with LTbR-Ig	3	3/3	184	184	184								
C57BL/6 treated with muIgG	3	3/3	184	184	184								
LTβR^−/−^	4	4/4	272	272	272	272							
CD40^−/−^	3	3/3	220	292	315								
C3^−/−^ C4^−/−^	3	3/3	363	363	420								
**intranasal inoculation**													
*Prnp* ^o/o^	8	0/8	>300	>300	>300	>300	>300	>300	>300	>300			
C57BL/6	8	8/8	219	219	253	263	292	292	292	296			
129SvxC57BL/6	5	5/5	187	213	213	235	235						
Balbc	6	6/6	112	225	225	225	225	242					
*tg*a*20*	10	10/10	118	125	126	133	152	165	186	187	202	203	
NSE-Prp	6	6/6	201	230	255	267	383	411					
Rag1^−/−^	9	9/9	198	198	198	200	203	203	204	210	214		
γ_C_Rag2^−/−^	16	16/16	224	224	224	229	241	242	242	242	244		
			244	256	258	264	265	265	319				
C1qa^−/−^	4	4/4	256	284	291	319							
CD21^−/−^	10	10/10	212	212	214	216	226	235	236	263	269	270	
CXCR5^−/−^	5	5/5	190	245	363	363	403						
C57BL/6 treated with LTβR-Ig	8	8/8	219	222	407	413	475	638	717	717			
C57BL/6 treated with muIgG	9	9/9	176	242	242	242	255	255	263	271	272		
LTβR^−/−^	6	6/6	223	252	263	314	346	348					
TNFR1^−/−^	3	3/3	213	213	214								
LTα^−/−^	6	6/6	233	234	238	255	262	283					
C57BL/6 HBH	4	0/4	>300	>300	>300	>300							
Balb/c HBH	4	0/4	>300	>300	>300	>300							
Rag1^−/−^ HBH	4	0/4	>300	>300	>300	>300							
γ_C_Rag2^−/−^ HBH	4	0/4	>300	>300	>300	>300							

### Prion aerosol infection of mice lacking LTβR or CD40L

LTβR signaling is essential for proper development of secondary lymphoid organs and for maintenance of lymphoid microarchitecture, and was recently shown to play an important role in prion replication within ectopic lymphoid follicles and granulomas [40], [41], [44]. To investigate the role of this pathway in aerogenic prion infections, *LTβR* ^−/−^ mice were exposed to prion aerosols (20% IBH; 10 min exposure time). All *LTβR* ^−/−^ mice succumbed to scrapie (*LTβR* ^−/−^: n = 4, 272±0 dpi) and displayed PrP deposits in their brains (Fig. 3C). Histological severity scoring of aerosol-exposed mice revealed higher scores in *LTβR* ^−/−^ hippocampi and lower scores in cerebellum, olfactory bulb, frontal and temporal white matter than in C57BL/6 controls (exposure: 20%; 10 min; Fig. 2E and 3C).

We then investigated the role of CD40 receptor in prion aerosol infection. *CD40* ^−/−^ mice fail to develop germinal centers and memory B-cell responses, yet *CD40L* ^−/−^ mice show unaltered incubation times upon i.p. prion challenge [54]. Similarly to the other immunocompromised mouse models investigated, *CD40* ^−/−^ mice developed terminal scrapie upon infection with prion aerosols with an attack rate of 100% (n = 3, 276±50 dpi). Lesion severity analyses of *CD40* ^−/−^ mice revealed a slightly higher score in the cerebellum and the temporal white matter than in C57BL/6 mice (Fig. 2E and 3C). Therefore, LTβR and CD40 signaling are dispensable for aerosolic prion infection.

### Components of the complement system are dispensable for aerosolic prion infection

Certain components of the complement system (e.g. C3; *C1q*a) play an important role in early prion uptake, peripheral prion replication and neuroinvasion after peripheral prion challenge [43], [55], [56]. We have tested whether this is true also for exposure to prion aerosols. Mice lacking both complement components C3 and C4 (*C3C4* ^−/−^) were exposed for 10 min to 20% aerosolized IBH. All *C3C4* ^−/−^ mice succumbed to scrapie (n = 3, 382±33 dpi; Fig. 4A). Histopathological evaluation of all scrapie affected mice revealed astrogliosis, spongiform changes and PrP-deposition in the CNS (Fig. 4A).

**Figure 4:** Prion transmission through aerosols in complement-deficient and newborn mice. (**A**) *C3C4* ^−/−^ mice and (**B**) newborn *tg*a*20* and CD1 mice were exposed for 10 min to a 20% aerosolized IBH. Survival curves **(right panels)** as well as histological and immunohistochemical characterization of hippocampi indicate that all prion-exposed mice developed scrapie efficiently. Scale bars: 100µm.

### No protection of newborn mice against prion aerosols

The data reported above argued in favor of direct neuroinvasion via PrP^C^-expressing neurons upon aerosol administration. However, a possible alternative mechanism of transmission may be via the ocular route, namely via cornea, retina, and optic nerve [57], [58]. In order to test this possibility, newborn (<24 hours-old) *tg*a*20* and CD1 mice, whose eyelids were still closed, were exposed for 10 min to prion aerosols generated from a 20% IBH. All mice succumbed to scrapie and showed PrP deposits in brains (*tg*a*20* mice: n = 3, 173±23 dpi; CD1 mice: n = 3, 211±0 dpi) (Fig. 4B). Newborn *tg*a*20* mice succumbed to scrapie slightly later (*p* = 0.0043) than adult *tg*a*20* mice, whereas no differences were observed between newborn and adult CD1 mice exposed for 10 min to prion aerosols generated from a 20% IBH (*p* = 0.392).

The brains of all animals contained PK-resistant material, as evaluated by Western blot analysis (data not shown). In addition, untreated littermates or other sentinels which were reared or housed together with aerosol-treated mice immediately following exposure to aerosols showed neither signs of scrapie nor PrP^Sc^ in brains, even after 482 dpi. This suggests that prion transmission was the consequence of direct exposure of the CNS to prion aerosols rather than the result of transmission via other routes like ingestion from fur by grooming or exposure to prion-contaminated feces or urine.

### Lack of PrP^Sc^ in secondary lymphoid organs of immunocompromised, scrapie-sick mice after infection with prion aerosols

We further investigated additional mice for the occurrence of PrP^Sc^ in secondary lymphoid organs upon exposure to prion aerosols. PK-resistant material was searched for in spleens, bronchial lymph nodes (bln) and mesenteric lymph nodes (mln) at terminal stage of disease. C57BL/6, 129SvxC57BL/6, muIgG treated C57BL/6 mice, newborn *tg*a*20* mice as well as newborn CD1 mice contained PrP^Sc^ in the LRS, whereas LTβR^−/−^ mice and C57BL/6 mice treated with LTβR-Ig lacked PrP^Sc^ deposits in spleens (Fig. S4A–F; Table 3).

**Table 3:** PrP^Sc^ deposition in spleens of mice challenged with a range of aerosolized prion concentrations and exposure times.

Genotype	Splenic PrP^Sc^ in individual mice										
	#1	#2	#3	#4	#5	#6	#7	#8	#9	#10	#11
*Prnp* ^o/o^	**−**	**−**	**−**								
Newborn CD1 (20%; 10 min exp.)	**+**	**+**	**+**								
CD1 (20%; 1 min exp.)	**+**	**+**	**+**	**+**	**−**	Nd	Nd				
CD1 (20%; 5 min exp.)	**+**	**+**	**−**	**−**	**+**	Nd	Nd				
CD1 (20%; 10 min exp.)	**+**	**+**	**+**	**+**	**+**	Nd	Nd	Nd			
C57BL/6 (20%; 10 min exp.)	**+**	**+**	**+**	**+**							
129SvxC57BL/6 (20%; 10 min exp.)	**+**	**+**	**+**	**+**	**+**						
Newborn *tg*a*20* (20%; 10 min exp.)	**+**	**+**	**+**								
*tg*a*20* (0.1%; 10 min exp.)	**−**	**−**	**−**	**−**							
*tg*a*20* (2.5%; 10 min exp.)	**+**	**+**	**+**	**+**							
*tg*a*20* (5%; 10 min exp.)	**+**	**+**	**+**	**+**							
*tg*a*20* (10%; 10 min exp.)	**+**	**+**	**+**	**+**	Nd						
*tg*a*20* (20%; 1 min exp.)	**+**	**+**	**+**	**+**	**−**	**−**					
*tg*a*20* (20%; 5 min exp.)	**+**	**+**	**+**	**+**	**+**	**+**	Nd	Nd			
*tg*a*20* (20%; 10 min exp.)	**+**	**+**	**+**	**+**	**+**	**+**	**+**	**+**			
*tg*a*20* (20%; 10 min exp.)	**+**	**+**	**+**	**+**	**+**	**+**	**+**				
JH^−/−^	**−**	**−**	**−**	**−**							
γ_C_Rag2^−/−^	**−**	**−**	**−**	**−**	**−**	**−**	**−**	**−**	**−**	**−**	**−**
C57BL/6 treated with LTβR-Ig	**−**	**−**	**−**								
C57BL/6 treated with mu-IgG	**+**	**+**	Nd								
LTβR^−/−^	**−**	**−**	**−**	**−**							

PrP^Sc^ was assessed on Western blots and histoblots of spleens of *Prnp* ^o/o^, newborn CD1, adult CD1, 129SvxC57BL/6, newborn *tg*a*20*, adult *tg*a*20*, JH^−/−^, γ_C_Rag2^−/−^, C57BL/6 mice treated with LTβR-Ig or muIgG and LTβR^−/−^ mice. +: PrP^Sc^ detectable in spleen; −: PrP^Sc^ undetectable; Nd: not determined; exp.: exposure time (minutes).

### The efficiency of intranasal prion inoculation depends on the level of PrP^C^ expression

To dissect aerosol-mediated from non-aerosolic contributions to prion exposure, we directly applied a prion suspension (RML 6.0, 0.1%, 40µl, corresponding to 4×10^5^ LD_50_ scrapie prions) to the nasal mucosa of various mouse lines (Fig. S5). Since mice breathe exclusively through their nostrils [59], [60] we reasoned that this procedure would simulate aerosolic transmission with sufficient faithfulness although the mechanisms of prion uptake could still differ between aerosolic and intranasal administration [11].

*tg*a*20* (n = 10), 129SvxC57BL/6 (n = 5), C57BL/6 (n = 8) and *Prnp* ^o/o^ mice (n = 8) were challenged intranasally with prions (Fig. S5). To test the possibility that the inoculation procedure itself might impact the life expectancy of mice, C57BL/6 mice (n = 4) were inoculated intranasally with healthy brain homogenate (HBH) for control (Fig. S5E). None of the animals that had been inoculated with HBH displayed a shortened life span, nor did they develop any clinical signs of disease - even when kept for ≥500 dpi. In contrast, after intranasal prion inoculation all C57BL/6, 129SvxC57BL/6 and *tg*a*20* mice succumbed to scrapie with an attack rate of 100% (Fig. S5A–C), whereas *Prnp* ^o/o^ mice were resistant to intranasal prions (Fig. S5D). After intranasal inoculation, *tg*a*20* mice (n = 10, 160±28 dpi) displayed a shorter incubation time (Fig. S5C) than 129SvxC57BL/6 (n = 5, 217±20 dpi) or C57BL/6 mice (n = 8, 266±33 dpi; Fig. S5A and S5B). Further, histological and immunohistochemical analyses for spongiosis, astrogliosis and PrP deposition pattern confirmed terminal scrapie (Fig. S5J). A histopathological lesion severity score analysis revealed similar lesion profiles as detected after exposure to prion aerosols (Fig. S5K). However, in the olfactory bulb of *tg*a*20* and 129SvxC57BL/6 mice the score was lower upon intranasal administration than in the aerosol paradigm (Fig. 2E).

Finally, we tested whether prion transmission via the intranasal route would be enabled by selective PrP^C^ expression on neurons. For that, we inoculated *NSE-PrP* mice. All intranasally challenged *NSE-PrP* mice (n = 6, 291±86 dpi) succumbed to scrapie. The incubation time until terminal disease did not differ significantly from that of 129SvxC57BL/6 control mice (n = 5, 217±20 dpi; *p* = 0.0868).

### Intranasal prion transmission in the absence of a functional immune system

Next, we sought to determine which components (if any) of the immune system are required for neuroinvasion upon intranasal infection with prions. To address this question, *Rag1* ^−/−^ and *γ_C_Rag2* ^−/−^ mice were intranasally inoculated with prions (inoculum RML 6.0, 0.1%, 40µl, equivalent to 4×10^5^ LD_50_ scrapie prions). Remarkably, all intranasally prion-inoculated *Rag1* ^−/−^ (n = 9, 203±6 dpi) (Fig. 5A and H) and *γ_C_Rag2* ^−/−^ mice (n = 16, 243±24 dpi) (Fig. 5D and G) succumbed to scrapie, providing evidence for a LRS-independent mechanism of prion neuroinvasion upon intranasal administration. Incubation times in *Rag1* ^−/−^ were significantly different to those of intranasally challenged control mice (C57BL/6; attack rate 100%; n = 8, 266±33 dpi; *p* = 0.0009) whereas *γ_C_Rag2* ^−/−^ mice were not different from those of intranasally challenged control mice (Balb/c: attack rate 100%, n = 6, 209±48 dpi, *p* = 0.099) (Fig. 5B and Fig. 5D).

**Figure 5:** Prion transmission by intranasal instillation. (**A**) *Rag1* ^−/−^ mice intranasally inoculated with RML6 0.1%, (**B**) C57BL/6 mice that have been intranasally inoculated with 3×10^5^ LD_50_ prions. (**C**) *Rag1* ^−/−^ mice i.c. inoculated with 3×10^5^ LD_50_, (**D**) *γ_C_Rag2* ^−/−^ mice intranasally inoculated with 4×10^5^ LD_50_ or (**E**) Balb/c mice intranasally inoculated with 4×10^5^ LD_50_ scrapie prions are shown. Survival curves (**A–D**) and respective Western blots (**F–G**) are indicative of efficient prion neuroinvasion. Brain homogenates were analyzed with (+) and without (−) previous proteinase K (PK) treatment as indicated. Brain homogenates derived from a terminally scrapie-sick and a healthy C57BL/6 mouse served as positive and negative controls (s: sick; h: healthy), respectively. Molecular weights (kDa) are indicated on the left side of the blots. (**H and I**) Histopathological lesion severity score described as radar blot (astrogliosis, spongiform change and PrP^Sc^ deposition) in 5 brain regions of both mouse lines exposed to prion aerosols. Numbers correspond to the following brain regions: (1) hippocampus, (2) cerebellum, (3) olfactory bulb, (4) frontal white matter, (5) temporal white matter.

After intranasal prion administration, PrP^Sc^ was present in the CNS of *Rag1* ^−/−^ or *γ_C_Rag2* ^−/−^ mice. WB analysis corroborated terminal scrapie (Fig. 5G and H). Histopathological lesion severity scoring revealed a distinct lesion profile characterized by a high score in the temporal white matter and the thalamus in case of *Rag1* ^−/−^ mice. In case of *γ_C_Rag2* ^−/−^ mice the cerebellum, the olfactory bulb and the frontal white matter displayed lower scores (Fig. 5I and J). In contrast to the CNS spleens of the affected animals did not contain PK-resistant material in terminally sick *Rag1* ^−/−^ and *γ_C_Rag2* ^−/−^ mice (Fig. S6E).

For control, Rag1^−/−^ as well as *γ_C_Rag2* ^−/−^ mice were intranasally inoculated with HBH to test the possibility that intranasal inoculation itself impacts their life expectancy. None of the mice inoculated with HBH died spontaneously or developed scrapie up to ≥300 dpi (n = 4 each; Fig. S6A, C–D). Further, Balb/c mice and C57BL/6 mice (n = 4 each) inoculated intranasally with HBH (Fig. S5E and S6D) did not develop any disease for ≥300 dpi.

As a positive control, *Rag1* ^−/−^ mice were i.c. inoculated with 3×10^5^ LD_50_ scrapie prions. This led to terminal scrapie disease after approximately 130 days and an attack rate of 100% (n = 3, 131±8 dpi) (Fig. 5B and data not shown).

As additional negative controls, *Rag1* ^−/−^ and *γ_C_Rag2* ^−/−^ mice were i.p. inoculated with prions (100 µl RML 0.1%, 1×10^6^ LD_50_). Although more infectious prions (approximately 2 fold more) were applied when compared to the intranasal route, i.p. prion inoculation did not suffice to induce scrapie in *Rag1* ^−/−^ and *γ_C_Rag2* ^−/−^ mice (attack rate: 0%, n = 4 for each group, experiment terminated after 400 dpi).

### Relevance of the complement system for prion pathogenesis after intranasal challenge

The complement component *C1q*a is involved in facilitating the binding of PrP^Sc^ to complement receptors on FDCs [56]. Accordingly, *C1q*a^−/−^ mice are resistant to prion infection upon low-dose peripheral inoculation. *CD21* ^−/−^ mice are devoid of the complement receptor 1, display a normal lymphoid microarchitecture and show a reduction in germinal center size. The incubation time in *CD21* ^−/−^ mice is greatly increased upon peripheral prion inoculation via the i.p. route [56].

To determine whether the complement system is involved in prion infection through aerosols, *C1q*a^−/−^ and *CD21* ^−/−^ mice were intranasally inoculated with prions. *C1q*a^−/−^ mice and *CD21* ^−/−^ mice succumbed to scrapie with an attack rate of 100% (*C1q*a^−/−^ mice: n = 4, 288±26 dpi; *CD21* ^−/−^ mice: n = 10, 235±24 dpi) (Figs. 6A–C), with *CD21* ^−/−^ mice succumbing to scrapie slightly earlier when compared to *C1q*a^−/−^ mice. However, survival times did not differ significantly from C57BL/6 control mice (n = 8, 266±33 dpi; *C1q*a^−/−^ mice: *p* = 0.24; *CD21* ^−/−^ mice: *p* = 0.05) (Fig. S5A and S5B). Western blot analysis of one terminally scrapie-sick *C1q*a^−/−^ mouse revealed one PrP^Sc^ positive spleen (1/4) (Fig. S6F). Two terminally scrapie-sick *CD21* ^−/−^ mice showed PK resistance in their spleens (2/10) (Fig. S6G). These results indicate that the complement components C1qa and CD21 are not essential for prion propagation upon intranasal application.

**Figure 6:** Intranasal prion transmission in immnunodeficient mice. All mice were intranasally inoculated with 3×10^5^ LD_50_ prions. (**A**) *C1q*a^−/−^ mice intranasally inoculated and (**B**) *CD21* ^−/−^ mice intranasally inoculated are shown. Survival curves illustrate survival after intranasal prion challenge. Respective Western blots of *C1qa* ^−/−^ mice intranasally inoculated (**C, left panel**) and of *CD21* ^−/−^ mice intranasally inoculated (**C, right panel**) are shown. Survival curves of *CXCR5* ^−/−^ mice intranasally inoculated are shown (**D**). Respective Western blots of *CXCR5* ^−/−^ mice intranasally inoculated. Brain homogenates were analyzed with (+) and without (−) previous proteinase K (PK) treatment as indicated. Controls and legends are as in Fig. 5.

### CXCR5 deficiency does not shorten prion incubation time upon intranasal infection

CXCR5 controls the positioning of B-cells in lymphoid follicles, and the FDCs of CXCR5-deficient mice are in close proximity to nerve terminals, leading to a reduced incubation time after i.p. prion inoculation [39], [61]. Here we explored the impact of CXCR5 deficiency onto intranasal prion inoculation. *CXCR5* ^−/−^ mice exhibited attack rates of 100%, and incubation times did not differ significantly from those of C57BL/6 mice (n = 5, 313±91 dpi; *p* = 0.32) (Fig. 6D). 3 out of 5 terminally scrapie-sick *CXCR5* ^−/−^ mice revealed PK resistant material in their spleens (3/5), as detected by Western blot analysis (Fig. S6H).

### Prion infection is independent of LTβR and TNFR1 signaling

Pharmacological inhibition of LTβR signaling strongly reduces peripheral prion replication and reduces or prevents prion neuroinvasion upon i.p. prion challenge [42], [44], [53]. To determine whether inhibition of LTβR signaling would affect prion transmission through the nasal cavity, we treated C57BL/6 mice with 100µg LTβR-Ig and for control with 100µg muIgG/mouse/week pre- and post-prion challenge (−7 days, 0 days, +7 days; 14 days). LTβR-Ig-treated mice were then inoculated intranasally with prions. 100% of the intranasally challenged mice died due to terminal scrapie (C57BL/6 mice treated with LTβR-Ig: n = 8, 476±200 dpi; Fig. 7A). MuIgG treated mice served as controls and showed an insignificantly shortened incubation time (attack rate: 100%, n = 9, 246±29 dpi) (Fig. 7B and C; C57BL/6 LTβR-Ig treated vs. muIgG treated mice: *p* = 0.014; C57BL/6 untreated vs. LTβR-Ig treated C57BL/6 mice: *p* = 0.021; C57BL/6 untreated vs. C57BL/6 muIgG treated mice: *p* = 0.22).

**Figure 7:** Intranasal prion transmission is independent of lymphotoxin signaling. C57BL/6 mice treated with LTβR-Ig (**A**) or control muIgG (**B**), and mice lacking various components of the LT/TNF system (**D–F**, as indicated) were intranasally inoculated with 4×10^5^ LD_50_ scrapie prions. Survival curves (**A, B, D, E** and **G**) and respective Western blots (**C, F** and **H**) indicate efficient prion infection and neuroinvasion. One animal that died early after intranasal inoculation (40 dpi) is reported as intercurrent death (i.d.) for reasons other than scrapie. Brain homogenates were analyzed with (+) and without (−) previous proteinase K (PK) treatment as indicated. Controls and legends used are as in Fig. 1H.

We additionally challenged *LTβR* ^−/−^, *TNFR1* ^−/−^ and *LTα* ^−/−^ mice intranasally with RML prions (Fig. 7D–H). Under these conditions all *LTβR* ^−/−^, *TNFR1* ^−/−^ *and LTα* ^−/−^ mice developed terminal scrapie (*LTβR* ^−/−^ mice: n = 6, 291±52 dpi; *TNFR1* ^−/−^ mice: n = 3, 213±1 dpi; *LTα* ^−/−^ mice: n = 6, 251±20 dpi) (Fig. 7D–H). Terminal scrapie was confirmed by immunohistochemistry, histoblot and WB analysis (Fig. 7F and H, data not shown). Spleens of intranasally inoculated *LTβR* ^−/−^ and *TNFR1* ^−/−^ mice displayed no PK resistant material (*LTβR* ^−/−^ mice: 0/6; *TNFR1* ^−/−^ mice: 0/3). In *LTα* ^−/−^ mice 1 out of 6 spleens contained PrP^Sc^, while splenic PrP^Sc^ deposits of PK-resistant material were abundantly found in terminally scrapie-sick *tg*a*20* mice (*tg*a*20* mice: 2/10)(Fig. S6I–L).

## Discussion

Although aerial transmission is common for many bacteria and viruses, it has not been thoroughly investigated for prion aerosols [11], [12], [29], [30], [31], [32], [33], [34], [62] and prions are not generally considered to be airborne pathogens. Yet olfactory nerves have been discussed as a possible entry site for prions [11], and indeed contact-mediated prion exposure of nostrils can efficiently infect various species. We therefore set out to investigate the possible hazards of prion infection deriving from exposure to prion aerosols. Our results establish that aerosolized prion-containing brain homogenates that aerosols are efficacious prion vectors.

Incubation time and attack rate after exposure to prion aerosols depended primarily on the exposure time, the PrP^C^ expression level of recipients and, to a lesser degree, the prion titer of the materials used to generate prion aerosols in a standardized inhalation chamber. The paramount role of the exposure time suggests that the rate of transepithelial ingress of prion through the airways may be limiting even when prions are offered in relatively low concentrations. Conversely, the total prion uptake capacity by the respiratory system was never rate-limiting, because the incubation time of scrapie decreased progressively with higher concentrations and longer exposure times, and because we were unable to establish a response plateau. The latter phenomenon may be explained by the large alveolar surface potentially available for prion uptake.

Since it occurred in wt mice of disparate genetic backgrounds (C57BL/6; CD1; 129SvxC57BL/6), aerosolic infection may represent a universal phenomenon untied to the genetic peculiarities of any specific mouse strain (Fig. S7 features a representative panel of histological features in CD1 mice). However, in CD1 mice the rapidity of progression to clinical disease did not correlate with the exposure time at a given concentration of IBH used for generating prion aerosols, suggesting the existence of genetic factors modulating the saturation of aerogenic prion intake.

The passage of infectivity from the peritoneum to the brain requires a non-hematopoietic conduit that expresses PrP^C^ [63]. We therefore sought to determine whether such a conduit would be required for transfer of infectivity from the aerosols to the brains of recipients. Using *NSE-PrP* transgenic mice, we found that neuron-selective expression of PrP^C^ sufficed to confer susceptibility of mice to prion infection by aerosols and intranasal application. Hence PrP^C^ expression in non-neural tissues is not required for aerosolic or intranasal neuroinvasion.

Following peripheral exposure, many TSE agents accumulate and replicate in host lymphoid tissues, including spleen, lymph nodes, Peyers' patches, and tonsils [59], [64], [65], [66], [67], [68], [69] in B-cell and lymphotoxin-dependent process [70], [71]. After peripheral replication in the LRS, prions gain access to the CNS primarily via peripheral nerves [23]; the innervation of secondary lymphoid organs and the distance between FDCs and splenic nerve endings is rate-limiting step for neuroinvasion [38] [39].

In contrast to the above, aerosolic and intranasal exposure led to prion infection in the absence of B-, T-, NK-cells and mature FDCs. Although a trend towards a slight delay in incubation time was detected in certain immunodeficient mice (e.g. LTβR^−/−^ and C3C4^−/−^) and after LTβR-Ig treatment, these differences were not statistically significant, and all other immunodeficient (*JH* ^−/−^, *Rag1* ^−/−^ and *γ_C_Rag2* ^−/−^) as well as complement-deficient (e.g. C3C4 and CD21) mice were susceptible to aerosolic and intranasal prion infection similarly to control mice. We conclude that transmission into the CNS upon aerosolic prion inoculation requires neither a functional adaptive immune system nor microanatomically intact germinal centers with mature FDCs. Further, the interference with LT signaling, be it by LTβR-Ig treatment or through ablation of the LTβR, indicates that the anatomical and functional intactness of lymphoid organs is dispensable for prion neuroinvasion, brain prion replication, and clinical scrapie.

Since genetic removal of the main cellular components of the LRS (e.g. by intercrosses with mice lacking T-, B-cells or NK-cells in, JH^−/−^ or γ_C_Rag2^−/−^ mice) as well as genetic (LTα^−/−^; LTβR^−/−^) or pharmacological (LTβR-Ig) depletion of follicular dendritic cells - the main cell responsible for prion replication in secondary lymphoid organs - did not change the course of disease upon infection with prion aerosols, we conclude that the above data demonstrate that the LRS is dispensable for prion infection through the aerogenic route. We therefore propose that airborne prions follow a pathway of direct prion neuroinvasion along olfactory neurons which extend to the surface of the olfactory epithelium. The infectibility of newborn mice supports this hypothesis, since these mice lacked a fully mature immune system at the time of prion exposure.

Our results contradict previous studies [12] claiming a role for the immune system in neuroinvasion upon intranasal prion infection, but are consistent with recent work [11] showing that prion neuroinvasion from the tongue and the nasal cavity can occur in the absence of a prion-infected LRS. Transmission of CWD to “cervidized” transgenic mice via aerosols and upon intranasal administration has also been shown [45].

Both *LTβR* ^−/−^ and *LTα* ^−/−^ mice lack Peyer's patches and lymph nodes as well as an intact NALT which may influence prion replication competence [11], [12], [29], [30], [31], [32], [33], [34], [63]. Furthermore, these mice display chronic interstitial pneumonia. Consistently with a role for LTβR-signaling in peripheral prion infection, these mice do not replicate intraperitoneally administered prions. On the other hand, *TNFR1* ^−/−^ mice lack Peyer's patches, show an aberrant splenic microarchitecture, an abnormal NALT, but have intact lymph nodes where prion replication can occur efficiently [72]. However, prion replication efficacy in spleen is almost completely abrogated [73] and *TNFR1* ^−/−^ mice die due to scrapie after a prolonged incubation time when peripherally challenged with prions.

In the present study, all LTα^−/−^ mice succumbed to scrapie upon intranasal infection, whereas some LTα^−/−^ mice acquired prion infection following nasal cavity exposure in a previous study [11]. The requirement for the LRS in intranasal prion infection may depend on the particular prion strain being tested and on the size of the administered inoculum. When present in sufficiently high titers, prions may be able to directly enter the nervous system via the nasal mucosa and olfactory nerve terminals (Fig. 8). However, at limiting doses, aerial prion infection may be potentiated by an LRS-dependent preamplification step (Fig. 8), e.g. in the bronchial lymph nodes (BLNs), the nose, the gut-associated lymphoid tissue (NALT; GALT), or the spleen. In this study, the particle size generated by the nebulizer ensured that the entire respiratory tract was flooded by the aerosol so that the prion-containing aerosolized brain homogenate would reach the alveolar surface of the lung. There, prions may also colonize airway-associated lymphoid tissues and gain access to the CNS (Fig. 8).

**Figure 8:** Model of the possible pathways of aerogenic prion transmission. **(left)** Prion aerosols entering the nasal cavity (1) may directly migrate through the nasal epithelium towards olfactory nerve terminals (2). Subsequently, prions reach olfactory bulb neurons and colonize the limbic system and other regions of the brain (3). Prions may be taken up by the eyes from where they could be transported via the visual system (e.g. optic nerves) to the CNS. O: olfactory system; V: visual system. Alternatively **(right)** prions may be taken up by immune cells residing in (1) the nasal cavity, the lung, or (2) the gastrointestinal tract, from where they may be transferred to lymphoreticular system (LRS) components such as bronchial lymph nodes (BALT), nasal associated lymphoid tissue (NALT), gastrointestinal lymphoid tissue (GALT), mesenteric lymph nodes, or spleen for further amplification. Subsequently, prions traffic towards peripheral nerve terminals (PNS), from where they invade the central nervous system (CNS). SC: spinal cord. Arrows indicate possible migration directions of prions once they have invaded the spinal cord.

Infection through conjunctival or corneal structures was not required, since newborn mice succumbed to scrapie with an incidence of 100% despite having closed eyelids. While newborn *tg*a*20*, but not CD-1, mice experienced slightly prolonged incubation times when compared to adult (6–8 week-old) mice of the same genotype, the anatomical structures of the nasopharynx (e.g. olfactory epithelium and olfactory nerves) are not similarly developed at postnatal day one when compared to adulthood, potentially leading to a less efficient prion uptake upon aerosol exposure (e.g. via olfactory nerves). Although unlikely, it can not be excluded that infection through conjunctival or corneal structures might contribute to a more efficient prion infection upon aerosol exposure. Be as it may, all newborn mice of either genotypes succumbed to terminal scrapie upon aerosol prion infection despite their lack of fully developed lymphoid organs, thereby bolstering our conclusion that the immune system is dispensable for prion transmission through aerosols.

In summary, our results establish aerosols as a surprisingly efficient modality of prion transmission. This novel pathway of prion transmission is not only conceptually relevant for the field of prion research, but also highlights a hitherto unappreciated risk factor for laboratory personnel and personnel of the meat processing industry. In the light of these findings, it may be appropriate to revise current prion-related biosafety guidelines and health standards in diagnostic and scientific laboratories being potentially confronted with prion infected materials. While we did not investigate whether production of prion aerosols in nature suffices to cause horizontal prion transmission, the finding of prions in biological fluids such as saliva, urine and blood suggests that it may be worth testing this possibility in future studies.

## Material and Methods

### Ethics statement

Animals were maintained under specific pathogen-free conditions and experiments were approved and conform to the guidelines of the Swiss Animal Protection Law, Veterinary office, Canton Zurich. Mouse experiments were performed under licenses 40/2002 and 30/2005 according to the regulations of the Veterinary office of the Canton Zurich and in accordance with the regulations of the Veterinary office Tübingen.

### Aerosols

Exposure of mice to aerosols was performed in inhalation chambers containing a nebulizer device (Art.No. 73-1963, Pari GmbH, Munich, Germany) run with a pressure of 1.5 bar generating 100% particles below 10 µm with 60% of the particles below 2.5 µm and 52% below 1.2 µm. Such particle sizes are considered to be able to reach upper and lower airways [74]. Prion infected material used throughout this study was RML6 strain obtained from the brains of diseased CD1 mice in its 6^th^ passage (RML6). Mice were exposed to aerosolized prion infected brain homogenates for one, five or ten minutes.

### Intracerebral prion inoculation of mice

*tg*a*20* mice serving as indicator mice were inoculated i.c. with brain tissue homogenate using 30 µl volumes (RML6 0.1%, 3×10^5^ LD_50_ scrapie prions). The animals were checked on a daily basis and were sacrificed when showing defined neurological signs such as severe gait disorders.

### Intranasal prion application in mice

Mice were anesthetized with Ketamine/Xylazin hydrochloride anaesthesia. 10 µl of RML6 (0.1%) were intranasally inoculated in each nostril and on the nasal epithelium by using a 10 µl pipette. The mice were held horizontally during inoculation process and for 1 minute following the inoculation. The whole procedure was repeated after a break of 20 minutes, reaching a final volume of 40 µl of RML6, 0.1% (4×10^5^ LD_50_ scrapie prions).

### Intraperitoneal prion application in mice

Mice were anesthetized with Ketamine/Xylazin hydrochloride anaesthesia. 100 µl of RML6 (0.1%) 1×10^6^ LD_50_ scrapie prions were i.p. inoculated into *Rag1* ^−/−^ and *γ_C_Rag2* ^−/−^ mice.

### Western blotting

Tissue homogenates were prepared in sterile 0.32 M sucrose using a Fast Prep FP120 (Savant, Holbrook, NY, USA) or a Precellys 24 (Bertin Technologies). For detection of PrP^Sc^ 15µl of a brain homogenate were digested with Proteinase K (30 µg/ml) and incubated for 30 min at 37°C. For detection of PrP^C^ no digestion was performed. Proteins were separated by SDS-PAGE and transferred to a PVDF (Immobilon-P, Millipore, Bedford, Mass., USA) or nitrocellulose membrane (Schleicher & Söhne). Prion proteins were detected by enhanced chemiluminescence (Western blotting reagent, Santa Cruz Biotechnology, Heidelberg, Germany) or ECL (from PerbioScience, Lausanne, CH), using mouse monoclonal anti-PrP antibody POM-1 and horseradish peroxidase (HRP) conjugated goat anti-mouse IgG1 antibody (Zymed).

### Histoblot analysis

Histoblots were performed as described previously [73]. Frozen brains that were cut into 12 µm-thick slices were mounted on nitrocellulose membranes. Total PrP, as well as PrP^Sc^ after digestion with 50 or 100 µg/ml proteinase K for 4 hrs at 37°C, were detected with the anti-prion POM1 antibody (1∶10000, NBT/BCIP, Roche Diagnostics).

### Histological analysis

Formalin-fixed tissues were treated with concentrated formic acid for 60 min to inactivate prion infectivity. Paraffin sections (2µm) and frozen sections (5 or 10µm) of brains were stained with hematoxylin/eosin. Antibodies GFAP (1∶300; DAKO, Carpinteris, CA) for astrocytes were applied and visualized using standard methods. Iba-1 (1∶1000; Wako Chemicals GmbH, Germany) was used for highlighting activated microglial cells. Postfixation in formalin was performed for ∼8 hrs and tissues were embedded in paraffin. After deparaffinisation, for PrP staining sections were incubated for 6 min in 98% formic acid and washed in distilled water for 30 min. Sections were heated to 100°C in a steamer in citrate buffer (pH 6.0) for 3 min, and allowed to cool down to room temperature. Sections were incubated in Ventana buffer and stains were performed on a NEXEX immunohistochemistry robot (Ventana instruments, Switzerland) using an IVIEW DAB Detection Kit (Ventana). After incubation with protease 1 (Ventana) for 16 min, sections were incubated with anti-PrP SAF-84 (SPI bio, A03208, 1∶200) for 32 min. Sections were counterstained with hematoxylin.

### Lesion profiling

We selected 5 anatomic brain regions from all investigated or at least 3 mice per experimental group. We evaluated spongiosis on a scale of 0–4 (not detectable, mild, moderate, severe and status spongiosus). Gliosis and PrP immunological reactivity was scored on a 0–3 scale (not detectable, mild, moderate, severe). A sum of the three scores resulted in the value obtained for the lesion profile for the individual animal. The ‘radar plots’ depict the scores for spongiform changes, gliosis and PrP deposition. Numbers correspond to the following brain regions: (1) hippocampus, (2) cerebellum, (3) olfactory bulb, (4) frontal white matter, (5) temporal white matter. Investigators blinded to animal identification performed histological analyses.

### Misfolded Protein Assay (MPA)

Misfolded Protein Assay (MPA) was performed as described previously [75]. The assay, which was performed on a 96-well plate is divided into two parts: the PSR1 Capture and an ELISA. For the PSR1 Capture the set up of each reaction was as following: 3µL of PSR1 beads (buffer removed) and 100µl of 1× TBSTT were spiked with brain homogenate, incubated at 37°C for 1hr with shaking at 750rpm, the beads were washed on the plate washer (ELX405 Biotek) 8 times with residual 50 µl/well TBST. Then 75µl/well of denaturing buffer was added. This was incubated at RT for 10min with shaking at 750rpm. Subsequently 30µl/well of neutralizing buffer were added. An additional incubation at RT for 5min with shaking at 750rpm followed. The beads were pulled down with a magnet. The ELISA was performed as follows: 150µL/well of the sample was transferred to an ELISA plate which was coated with POM19. An incubation step at 37°C for 1hr with shaking at 300rpm followed. That was washed 6 times with wash buffer. POM2-AP conjugate had to be diluted to 0.01µg/mL in conjugate diluent. 150µL/well of diluted conjugate was added. Incubation at 37°C for 1hr without shaking followed. Washing 6 times with wash buffer was followed by preparation of enhanced substrate by adding 910µL of enhancer to 10mL of substrate (Lumiphos plus, Lumigen). 150µL/well of enhanced substrate was added. Incubation at 37°C for 30min was followed by reading by luminometer (Luminoskan Ascent) at default PMT, filter scale = 1.

### Real-time RT-PCR for quantification of the transgene copy number in *Prnp* ^o/o^/*NSE-PrP* mice

Real-time PCR was performed on purified genomic DNA from mouse tails on a 7900 HT Fast Real-Time PCR System (AB). Data were generated and analyzed using SDS 2.3 and RQ manager 1.2 software. The following primers were used: Forward primer annealing in mouse *Prnp* gene intron 1: 5′ - GGT TTG ATG ATT TGC ATA TTA G - 3′. Reverse primer annealing in mouse *Prnp* gene exon 2: 5′ - GGA AGG CAG AAT GCT TCA GC - 3′. The PCR product is approximately 200 bps in length. For control, the mouse Lymphotoxin alpha gene was analyzed. The following primers were used: Forward primer annealing to the Exon 1 of the mouse Lymphotoxin alpha gene: 5′ - CCT GGT GAC CCT GTT GTT GG - 3′. Reverse primer annealing to the mouse Lymphotoxin alpha gene Intron 1: 5′ - GTG GGC AGA AGC ACA GCC - 3′. The PCR product is approximately 160 bps in lenght. Real time PCR analysis revealed 2–4 transgene copies per *Prnp* allele in *Prnp* ^o/o^ */NSE-PrP* mice.

### Statistical evaluation

Results are expressed as the mean+standard error of the mean (SEM) or standard deviation (SD) as indicated. Statistical significance between experimental groups was assessed using an unpaired two-sample Student's t-Test (Excel) and two-sample Welch t-Test for distributions with unequal variance (R). For survival analyses, Kaplan-Meier-survival curves were generated using SPSS or R software, statistical significance was assessed by performing log rank tests (R). Linear regression fits and analyses of variance (ANOVA) were conducted in R (www.r-project.org).

## Supporting Information

Figure S1 Analysis of variance (ANOVA) for various genotypes regarding incubation times.
Dot plot of survival times for *tg*a*20*, CD1, C57BL/6 and 129SvxC57BL/6 mice after 10 min exposure to IBH. The difference between genotypes is significant (p<0.001).
(0.14 MB TIF)

Figure S2 Prion transmission through aerosols or upon intranasal challenge cannot be directly followed by Western blot and PMA.
(**A–D**) Western blot analysis for PrP^Sc^ of the compartments olfactory epithelium (OE), olfactory bulb (OB), one brain hemisphere or the cerebellum at 60 days post aerosolic infection in different mouse strains (C57BL/6, CXCR5^−/−^, CD21^−/−^, *Prnp* ^o/o^, CD1, LTα^−/−^, *NSE-PrP*, TNFR1^−/−^ mice). (+) and without (−) previous proteinase K (PK) treatment as indicated. Molecular weights (kDa) are indicated on the right side of the blots. kDa: Kilo Dalton. β-Actin served as a loading control. (**E**) Analysis of brain tissue homogenates from intranasally inoculated mice by the “misfolded protein assay” (MPA) reveals positive signals as indicators of Prp^Sc^ deposition in the control specimen (red) and negative signal in most cases investigated (blue, below wt level). The brain of a wt mouse was used as control (black). Y-axis: RLU: Relative (Chemi) Luminescence Units, X-axis: mouse number, blue column represents a 1∶10 dilution of a 10% brain homogenate. Data for uninfected brain controls are not shown here, but did not display a positive signal. (**F**) Analysis of olfactory bulb tissue homogenates from intranasally inoculated mice by the “misfolded protein assay” (MPA) reveals positive signals as indicators of Prp^Sc^ deposition in the control specimen (red) and in diseased mice (positive signals). Negative signals in most other cases investigated (blue bars under wt control level). The brain of a wt mouse was used as control (black). Y-axis: RLU: Relative (Chemi) Luminescence Units, X-axis: mouse number, blue column represents a 1∶10 dilution of a 10% brain homogenate. Data for uninfected brain controls are not shown here, but did not display a positive signal.
(0.68 MB TIF)

Figure S3 Detailed quantitative analysis of PrP^C^ expression in the olfactory epithelium and the CNS.
(**A**) Quantification of PrP^C^ expression levels by Western blotting in *NSE-PrP*, wt and *tg*a*20* mice. In the olfactory epithelium *tg*a*20* mice ≥3.5 fold higher PrP^C^ expression compared to wt mice and approximately 11 fold higher PrP^C^ expression compared to *NSE-PrP* mice. (**B**) In the olfactory bulb of *tg*a*20* mice ≥1.5 fold higher PrP^C^ expression compared to wt mice and more than 3.5 fold higher PrP^C^ expression compared to *NSE-PrP* mice. (**C**) In brain hemispheres of *tg*a*20* mice more than 2.5 fold higher PrP^C^ expression compared to wt mice, and more than 1.5 fold higher PrP^C^ expression compared to *NSE-PrP* mice. Molecular weights (kDa) are indicated on the right side of the blots. kDa: Kilo Dalton. β-Actin served as a loading control.
(1.48 MB TIF)

Figure S4 Splenic involvement after prion transmission through aerosols and involvement of the spleen.
(**A**) *tg*a*20* mice, (**B**) JH^−/−^ mice, (**C**) LTβR^−/−^ mice and (**D**) *γ_C_Rag2* ^−/−^ mice in part show splenic deposits of PK resistant material, evaluated by Western blot analysis. (**E**) Histoblot analysis of spleens of C57BL/6, of *Prnp* ^o/o^ and of *Rag1* ^−/−^ mice. C57BL/6 mice reveal PK resistant deposits while *Prnp* ^o/o^ and *Rag1* ^−/−^ mice lack such deposits. (**F**) Western blot analysis of a representative *tg*a*20* spleen, mesenteric lymph node (mln) and bronchial lymph node (bln) lacking PK-resistant material. (+) and (−) with or without PK treatment. POM1 was used as primary antibody.
(2.81 MB TIF)

Figure S5 Prion transmission via the intranasal route.
Survival curves of (**A**) C57BL/6, (**B**) 129SvxC57BL/6 (**C**) *tg*a*20* and (**D**) *Prnp* ^o/o^ mice that have been intranasally inoculated with RML6 0.1%. (**E**) Survival curve of C57BL/6 mice that have been intranasally inoculated with HBH. Western blots of brains of (**F**) C57BL/6 mice and of (**G**) *tg*a*20* mice that have been intranasally inoculated with 4×10^5^ LD_50_ scrapie prions. Brain homogenates were analyzed with (+) and without (−) previous proteinase K (PK) treatment as indicated. Homogenate derived from a terminally scrapie-sick mouse served as positive control (s: sick), and healthy C57BL/6 mouse brain homogenate as negative control (h: healthy), respectively. Molecular weights (kDa) are indicated on the left side of the blots. (**H**) Survival curves of *NSE-PrP* mice intranasally inoculated with prions are shown **(left panel)**. Respective Western blots of *NSE-PrP* mice intranasally inoculated with prions are shown **(right panel)**. Brain homogenates were analyzed with (+) and without (−) previous proteinase K (PK) treatment as indicated. Homogenate derived from a terminally scrapie-sick mouse served as positive control (s: sick), and healthy C57BL/6 mouse tissue as negative control (h: healthy), respectively and i.d. indicates intercurrent death of animal. Molecular weights (kDa) are indicated on the left side of the blots. (**I**) Histoblot analysis of prion infected mouse brains. Left panel: shows healthy brain of a *Prnp* ^o/o^ mouse as negative control, other panels demonstrate Prp^Sc^ deposits in brains of *tg*a*20* mice. Scale bars are indicated. (**J**) Histological and immunohistochemical characterization of scrapie affected mouse brains. Brain sections of *Prnp* ^o/o^, *tg*a*20*, 129SvxC57BL/6 and C57BL/6 mice as evaluated by HE (for spongiosis, gliosis, neuronal cell loss), SAF84 (for PrP^Sc^ deposits), GFAP (for astrogliosis) and Iba-1 (for microglial activation). Scale bars: 100µm. (**K**) Histopathological lesion severity score of 5 brain regions described as radar blot (astrogliosis, spongiform change and PrP^Sc^ deposition) of intranasally prion inoculated *tg*a*20*, C57BL/6 and 129SvxC57BL/6 mice.
(1.04 MB TIF)

Figure S6 Prion transmission via the intranasal route, controls and involvement of the spleen.
(**A**) *Rag1* ^−/−^ mice intranasally inoculated with HBH (40 µl) or (**B**) C57BL/6 intranasally inoculated with 4×10^5^ LD_50_ scrapie prions. (**C**) *γ_C_Rag2* ^−/−^ mice intranasally inoculated with HBH (40 µl) or (**D**) Balb/c mice intranasally inoculated with HBH are shown. Kaplan-Meier curves describe the percentage of survival after particular time points post intranasal prion inoculation (y-axis represents percentage of living animals; x-axis demonstrates survival time in days). Respective Western blots of (**E**) spleens and bln of terminal *Rag1* ^−/−^ mice, (**F**) of spleens of terminal C1q*a* ^−/−^ mice, (**G**) spleens of terminal CD21^−/−^ mice, (**H**) spleens of terminal CXCR5^−/−^ mice, (**I**) spleens of terminal LTβR^−/−^ mice, (**J**) spleens of terminal TNFR1^−/−^ mice, (**K**) spleens of terminal LTα^−/−^ and LTβR^−/−^ mice and (**L**) spleens of terminal *tg*a*20* mice.
(1.41 MB TIF)

Figure S7 Histological, immunohistochemical and immunoblot confirmation of prion disease upon aerosol infection.
(**A, B**) Histological and immunohistochemical characterization of scrapie affected CD1 mouse brains. (**A**) Representative olfactory bulbs (HE and Neurofilament stains) are shown. scale bars indicated (**B**) The cerebellum (upper row), the midbrain (second row from top), the frontal cortex (third row from top) and the olfactory bulb (lower row) display spongiosis, astrogliosis, microglial activation and Prp^Sc^ deposits upon prion infection via aerosols (HE, GFAP, Iba-1 and SAF-84 staining). Scale bars: 50 γm.
(8.63 MB TIF)

Table S1 **Survival times of mouse strains exposed to prion aerosols for various periods.**
(**A**) Analysis of variance for plates in Fig. 1F–G and Fig. S1. The time of exposure to aerosolized infectious brain homogenates, but not their concentration, significantly correlated with survival time. (**B**) Linear regression fits for survival time against exposure time in *tg*a*20* (Fig. 1G) and CD1 (Fig. S1) mice. Incubation times correlated negatively with PrP expression level. (**C**) Pair wise tests for differing mean survival time for *tg*a*20*, CD1, C57BL/6 and 129SvxC57BL/6 mice after 10 minutes exposure to prion aerosols (Fig. S1), identifying *Prnp* gene copy number as the strongest independent variable. *P*<0.001: ***, *P*<0.01: **, *P*<0.05: *, *P*<0.1.
(0.06 MB DOC)

## References

[1] Prusiner SB (1998). Prions.. Proc Natl Acad Sci U S A.

[2] Will RG (1999). Prion related disorders.. J R Coll Physicians Lond.

[3] Cuille J, Chelle PL (1939). Experimental transmission of trembling to the goat.. C R Seances Acad Sci.

[4] Weissmann C, Enari M, Klohn PC, Rossi D, Flechsig E (2002). Transmission of prions.. J Infect Dis.

[5] Hill AF, Desbruslais M, Joiner S, Sidle KC, Gowland I (1997). The same prion strain causes vCJD and BSE.. Nature.

[6] Maignien T, Lasmezas CI, Beringue V, Dormont D, Deslys JP (1999). Pathogenesis of the oral route of infection of mice with scrapie and bovine spongiform encephalopathy agents.. J Gen Virol.

[7] Heppner FL, Christ AD, Klein MA, Prinz M, Fried M (2001). Transepithelial prion transport by M cells.. Nat Med.

[8] Herzog C, Sales N, Etchegaray N, Charbonnier A, Freire S (2004). Tissue distribution of bovine spongiform encephalopathy agent in primates after intravenous or oral infection.. Lancet.

[9] Zhang J, Chen L, Zhang BY, Han J, Xiao XL (2004). Comparison study on clinical and neuropathological characteristics of hamsters inoculated with scrapie strain 263K in different challenging pathways.. Biomed Environ Sci.

[10] Aguzzi A, Polymenidou M (2004). Mammalian prion biology: one century of evolving concepts.. Cell.

[11] Bessen RA, Martinka S, Kelly J, Gonzalez D (2009). Role of the lymphoreticular system in prion neuroinvasion from the oral and nasal mucosa.. J Virol.

[12] Sbriccoli M, Cardone F, Valanzano A, Lu M, Graziano S (2009). Neuroinvasion of the 263K scrapie strain after intranasal administration occurs through olfactory-unrelated pathways.. Acta Neuropathol.

[13] Mathiason CK, Powers JG, Dahmes SJ, Osborn DA, Miller KV (2006). Infectious prions in the saliva and blood of deer with chronic wasting disease.. Science.

[14] Seeger H, Heikenwalder M, Zeller N, Kranich J, Schwarz P (2005). Coincident scrapie infection and nephritis lead to urinary prion excretion.. Science.

[15] Vascellari M, Nonno R, Mutinelli F, Bigolaro M, Di Bari MA (2007). PrPSc in Salivary Glands of Scrapie-Affected Sheep.. J Virol.

[16] Tamguney G, Miller MW, Wolfe LL, Sirochman TM, Glidden DV (2009). Asymptomatic deer excrete infectious prions in faeces.. Nature.

[17] Lacroux C, Simon S, Benestad SL, Maillet S, Mathey J (2008). Prions in milk from ewes incubating natural scrapie.. PLoS Pathog.

[18] Dickinson AG, Stamp JT, Renwick CC (1974). Maternal and lateral transmission of scrapie in sheep.. J Comp Pathol.

[19] Foster J, McKenzie C, Parnham D, Drummond D, Chong A (2006). Lateral transmission of natural scrapie to scrapie-free New Zealand sheep placed in an endemically infected UK flock.. Vet Rec.

[20] Foster J, McKenzie C, Parnham D, Drummond D, Goldmann W (2006). Derivation of a scrapie-free sheep flock from the progeny of a flock affected by scrapie.. Vet Rec.

[21] Miller MW, Williams ES (2003). Prion disease: horizontal prion transmission in mule deer.. Nature.

[22] Ryder S, Dexter G, Bellworthy S, Tongue S (2004). Demonstration of lateral transmission of scrapie between sheep kept under natural conditions using lymphoid tissue biopsy.. Res Vet Sci.

[23] Aguzzi A, Heikenwalder M (2006). Pathogenesis of prion diseases: current status and future outlook.. Nat Rev Microbiol.

[24] Hadlow WJ, Kennedy RC, Race RE (1982). Natural infection of Suffolk sheep with scrapie virus.. J Infect Dis.

[25] Miller MW, Williams ES, Hobbs NT, Wolfe LL (2004). Environmental sources of prion transmission in mule deer.. Emerg Infect Dis.

[26] Bartz JC, Kincaid AE, Bessen RA (2003). Rapid prion neuroinvasion following tongue infection.. J Virol.

[27] Zanusso G, Ferrari S, Cardone F, Zampieri P, Gelati M (2003). Detection of pathologic prion protein in the olfactory epithelium in sporadic Creutzfeldt-Jakob disease.. N Engl J Med.

[28] Tabaton M, Monaco S, Cordone MP, Colucci M, Giaccone G (2004). Prion deposition in olfactory biopsy of sporadic Creutzfeldt-Jakob disease.. Ann Neurol.

[29] Kincaid AE, Bartz JC (2007). The nasal cavity is a route for prion infection in hamsters.. J Virol.

[30] DeJoia C, Moreaux B, O'Connell K, Bessen RA (2006). Prion infection of oral and nasal mucosa.. J Virol.

[31] Doty RL (2008). The olfactory vector hypothesis of neurodegenerative disease: is it viable?. Ann Neurol.

[32] Corona C, Porcario C, Martucci F, Iulini B, Manea B (2009). Olfactory system involvement in natural scrapie disease.. J Virol.

[33] Hamir AN, Kunkle RA, Richt JA, Miller JM, Greenlee JJ (2008). Experimental transmission of US scrapie agent by nasal, peritoneal, and conjunctival routes to genetically susceptible sheep.. Vet Pathol.

[34] Park CH, Ishinaka M, Takada A, Kida H, Kimura T (2002). The invasion routes of neurovirulent A/Hong Kong/483/97 (H5N1) influenza virus into the central nervous system after respiratory infection in mice.. Arch Virol.

[35] Shaw IC (1995). BSE and farmworkers [letter].. Lancet.

[36] Sawcer SJ, Yuill GM, Esmonde TF, Estibeiro P, Ironside JW (1993). Creutzfeldt-Jakob disease in an individual occupationally exposed to BSE.. Lancet.

[37] Reuber M, Al-Din AS, Baborie A, Chakrabarty A (2001). New variant Creutzfeldt-Jakob disease presenting with loss of taste and smell.. J Neurol Neurosurg Psychiatry.

[38] Glatzel M, Heppner FL, Albers KM, Aguzzi A (2001). Sympathetic innervation of lymphoreticular organs is rate limiting for prion neuroinvasion.. Neuron.

[39] Prinz M, Heikenwalder M, Junt T, Schwarz P, Glatzel M (2003). Positioning of follicular dendritic cells within the spleen controls prion neuroinvasion.. Nature.

[40] Heikenwalder M, Zeller N, Seeger H, Prinz M, Klohn PC (2005). Chronic lymphocytic inflammation specifies the organ tropism of prions.. Science.

[41] Heikenwalder M, Kurrer MO, Margalith I, Kranich J, Zeller N (2008). Lymphotoxin-dependent prion replication in inflammatory stromal cells of granulomas.. Immunity.

[42] Mabbott NA, Young J, McConnell I, Bruce ME (2003). Follicular dendritic cell dedifferentiation by treatment with an inhibitor of the lymphotoxin pathway dramatically reduces scrapie susceptibility.. J Virol.

[43] Mabbott NA, Bruce ME, Botto M, Walport MJ, Pepys MB (2001). Temporary depletion of complement component C3 or genetic deficiency of C1q significantly delays onset of scrapie.. Nat Med.

[44] Mabbott NA, Mackay F, Minns F, Bruce ME (2000). Temporary inactivation of follicular dendritic cells delays neuroinvasion of scrapie.. Nat Med.

[45] Denkers ND, Seelig DM, Telling GC, Hoover EA (2010). Aerosol and nasal transmission of chronic wasting disease in cervidized mice.. J Gen Virol.

[46] Fischer M, Rülicke T, Raeber A, Sailer A, Moser M (1996). Prion protein (PrP) with amino-proximal deletions restoring susceptibility of PrP knockout mice to scrapie.. EMBO J.

[47] Radovanovic I, Braun N, Giger OT, Mertz K, Miele G (2005). Truncated prion protein and Doppel are myelinotoxic in the absence of oligodendrocytic PrPC.. J Neurosci.

[48] Sigurdson CJ, Nilsson KP, Hornemann S, Heikenwalder M, Manco G (2009). De novo generation of a transmissible spongiform encephalopathy by mouse transgenesis.. Proc Natl Acad Sci U S A.

[49] Sigurdson CJ, Nilsson KP, Hornemann S, Manco G, Polymenidou M (2007). Prion strain discrimination using luminescent conjugated polymers.. Nat Methods.

[50] Radovanovic I, Braun N, Giger OT, Mertz K, Miele G (2005). Truncated Prion Protein and Doppel Are Myelinotoxic in the Absence of Oligodendrocytic PrPC.. J Neurosci.

[51] Montrasio F, Frigg R, Glatzel M, Klein MA, Mackay F (2000). Impaired prion replication in spleens of mice lacking functional follicular dendritic cells.. Science.

[52] Mackay F, Browning JL (1998). Turning off follicular dendritic cells.. Nature.

[53] Huber C, Thielen C, Seeger H, Schwarz P, Montrasio F (2005). Lymphotoxin-beta receptor-dependent genes in lymph node and follicular dendritic cell transcriptomes.. J Immunol.

[54] Heikenwalder M, Federau C, Boehmer L, Schwarz P, Wagner M (2007). Germinal center B cells are dispensable in prion transport and neuroinvasion.. J Neuroimmunol.

[55] Zabel MD, Heikenwalder M, Prinz M, Arrighi I, Schwarz P (2007). Stromal complement receptor CD21/35 facilitates lymphoid prion colonization and pathogenesis.. J Immunol.

[56] Klein MA, Kaeser PS, Schwarz P, Weyd H, Xenarios I (2001). Complement facilitates early prion pathogenesis.. Nat Med.

[57] Wadsworth JDF, Joiner S, Hill AF, Campbell TA, Desbruslais M, Luthert PJ, Collinge J (2001). Tissue distribution of protease resistant prion protein in variant CJD using a highly sensitive immuno-blotting assay.. Lancet.

[58] Safar J, Wille H, Itri V, Groth D, Serban H (1998). Eight prion strains have PrP(Sc) molecules with different conformations.. Nat Med.

[59] Agrawal A, Singh SK, Singh VP, Murphy E, Parikh I (2008). Partitioning of nasal and pulmonary resistance changes during noninvasive plethysmography in mice.. J Appl Physiol.

[60] Bates JH, Irvin CG (2003). Measuring lung function in mice: the phenotyping uncertainty principle.. J Appl Physiol.

[61] Aguzzi A, Heikenwalder M, Miele G (2004). Progress and problems in the biology, diagnostics, and therapeutics of prion diseases.. J Clin Invest.

[62] Diringer H (1995). Proposed link between transmissible spongiform encephalopathies of man and animals.. Lancet.

[63] Blättler T, Brandner S, Raeber AJ, Klein MA, Voigtländer T (1997). PrP-expressing tissue required for transfer of scrapie infectivity from spleen to brain.. Nature.

[64] Sigurdson CJ, Williams ES, Miller MW, Spraker TR, O'Rourke KI (1999). Oral transmission and early lymphoid tropism of chronic wasting disease PrPres in mule deer fawns (Odocoileus hemionus).. J Gen Virol.

[65] Hilton DA, Fathers E, Edwards P, Ironside JW, Zajicek J (1998). Prion immunoreactivity in appendix before clinical onset of variant Creutzfeldt-Jakob disease. Lancet.

[66] Mabbott NA, MacPherson GG (2006). Prions and their lethal journey to the brain.. Nat Rev Microbiol.

[67] Hill AF, Zeidler M, Ironside J, Collinge J (1997). Diagnosis of new variant Creutzfeldt-Jakob disease by tonsil biopsy.. Lancet.

[68] Mould DL, Dawson AM, Rennie JC (1970). Very early replication of scrapie in lymphocytic tissue.. Nature.

[69] Beekes M, McBride PA (2000). Early accumulation of pathological PrP in the enteric nervous system and gut-associated lymphoid tissue of hamsters orally infected with scrapie.. Neurosci Lett.

[70] Klein MA, Frigg R, Raeber AJ, Flechsig E, Hegyi I (1998). PrP expression in B lymphocytes is not required for prion neuroinvasion.. Nat Med.

[71] Klein MA, Frigg R, Flechsig E, Raeber AJ, Kalinke U (1997). A crucial role for B cells in neuroinvasive scrapie.. Nature.

[72] Prinz M, Montrasio F, Klein MA, Schwarz P, Priller J (2002). Lymph nodal prion replication and neuroinvasion in mice devoid of follicular dendritic cells.. Proc Natl Acad Sci U S A.

[73] Taraboulos A, Jendroska K, Serban D, Yang SL, DeArmond SJ (1992). Regional mapping of prion proteins in brain.. Proc Natl Acad Sci U S A.

[74] Raab OG, Yeh HC, Newton GJ, Phalen RF, Velasquez DJ (1975). Deposition of inhaled monodisperse aerosols in small rodents.. Inhaled Part.

[75] Lau AL, Yam AY, Michelitsch MM, Wang X, Gao C (2007). Characterization of prion protein (PrP)-derived peptides that discriminate full-length PrPSc from PrPC.. Proc Natl Acad Sci U S A.

